RETRACTED

# Simvastatin in the Treatment of Colorectal Cancer: A Review

**DOI:** 10.1155/2022/3827933

**Published:** 2022-07-14

**Authors:** Hongliang Zang, Wei Yang, Xiaofeng Tian

**Affiliations:** Department of Hepatopancreatobiliary Surgery, China-Japan Union Hospital of Jilin University, Changchun, China

## Abstract

Drug repositioning and drug reuse are the heated topics in the field of oncology in recent years. These two concepts refer to seeking effective drugs for cancer that are not originally intended to treat cancer. The survival benefits are then analyzed by combining the re-positioned drugs with conventional cancer treatment methods. Simvastatin is a clinically commonly used hyperlipidemia drug and exerts the effect of preventing cardiovascular diseases. Recent studies have found that simvastatin has great potential in the treatment of colorectal cancer, and a large number of clinical studies have used simvastatin as an adjuvant drug to help treat metastatic colorectal cancer.

## 1. Introduction

Colorectal cancer is one of the most common malignant tumors worldwide, with the incidence ranking third among all malignant tumors, and the mortality ranking second [1, 2]. The WHO Cancer Research Centre's GLOBOCAN project estimated that the number of new colorectal cancer cases worldwide in 2018 was approximately 1.8 million and the number of deaths was approximately 880,000 [3]. The incidence of colorectal cancer is related to age, region, and gender, with colorectal cancer mainly occurring in middle-aged and elderly people over 40 years of age [3]. In recent years, the incidence and mortality rate of colorectal cancer in China have been on the rise, which should be given sufficient attention. Due to the large individual differences, there is no absolute best, fastest, and most effective medication. Apart from the commonly used over-the-counter drugs, the most suitable drug should be selected under the guidance of a doctor, taking into full consideration the individual situation. The main drug treatments for colorectal cancer are targeted drugs, bevacizumab and cetuximab [4]. Bevacizumab binds to the vascular endothelial growth factor (VEGF) and inhibits proliferation and neovascularisation of tumour endothelium, reducing tumour tissue nutrition and thus may inhibit tumour growth [5]. Cetuximab is recommended for patients with wild-type K-ras, N-ras, and BRAF genes, and it inhibits the proliferation of cancer cells and induces apoptosis by blocking intracellular signaling pathways through binding to the epidermal growth factor (EGF) receptor [6]. The use of cetuximab in combination with radiotherapy and cisplatin has been associated with increased serious adverse events, such as cardiac events, compared to radiotherapy and cisplatin alone [7]. Despite the clinical advantages of immunotherapy, it is available for a specific population, and the drug option for sudden aggravated colorectal cancer in the course of treatment is limited [8, 9].

RETRACTED

Considering the high cost of expense and time to develop new drugs in clinical practice, some scholars proposed the flexible and economical concepts of drug repositioning and drug reuse. Statins, 3-hydroxy-3-methylglutaraldehyde coenzyme A (HMG-CoA) reductase inhibitors, can effectively prevent the conversion of HMG-CoA into meglutarate, thereby reducing the synthesis of cholesterol in patients [10, 11]. Statins are commonly used drugs to treat hyperlipidemia and prevent cardiovascular diseases. In recent years, relevant studies have pointed out that statins have good therapeutic effects on a variety of diseases, including cancer, through their involvement in angiogenesis, proliferation, apoptosis, and metastasis pathways [12, 13]. Furthermore, studies have shown that among statins, simvastatin, which has high lipophilicity, shows a beneficial anticancer activity in colon cancer cell lines. Furthermore, some studies have shown that simvastatin is effective in reducing the risk of colorectal cancer in patients. Many clinical trials have begun to add simvastatin to colorectal cancer chemotherapy regimens for the treatment of patients with metastatic colorectal cancer [14–17]. This article reviews the possible mechanisms of action of simvastatin in the treatment of colorectal cancer and the current status of its use in relevant clinical trials.

## 2. Analysis of the Possible Mechanism of Simvastatin in the Treatment of Colorectal Cancer

### 2.1. Simvastatin Combined with Cetuximab for KRAS-Mutated Colorectal Cancer

The colorectal cancer diagnostic guidelines (Chinese Society of Clinical Oncology) do not recommend the EGRF inhibitor cetuximab for KRAS-mutated colorectal cancer patients [18]. Kodach et al. (2011) also pointed out that the EGRF inhibitor cetuximab is not effective in the treatment of KRAS-mutated colorectal cancer patients [19]. Because KRAS is a key part of the EGFR signaling pathway, a mutation in the KRAS gene would make it insensitive to EGFR signaling and thus affect the effectiveness of EGFR inhibitors. Simvastatin is an (HMG-CoA) reductase inhibitor that interferes with the production of derivatives of the mevalonate pathway: farnesyl pyrophosphate and geranyl pyrophosphate. They are important substrates for Ras and Rho and play a key role in cell growth, proliferation, migration, and intracellular signaling [20]. Simvastatin can interfere with the Ras function, inhibit downstream signal transduction pathways (inhibit BRAF enzyme activity), and reverse cetuximab resistance in KRAS-mutant colorectal cancer cell lines.

RETRACTED

### 2.2. The Antiangiogenesis Effect of Simvastatin on Colorectal Cancer

New blood vessels can supply energy and oxygen to cancer cells and also have a role in tumor metastasis. Tumor angiogenesis is regulated by various cytokines in the tumor microenvironment. The vascular endothelial growth factor is overexpressed in most cancer cells, which makes it the main target of the cancer antiangiogenic therapy. The overexpression of human epidermal growth factor receptor 2 promotes tumor angiogenesis. The vascular endothelial growth factor, human epidermal growth factor receptor 2, and phosphorylated human epidermal growth factor receptor 2 are consistently expressed at high levels in colorectal cancer patient cells. Among animal experiments, Lee et al. (2009) found that the expression of oncogenic human epidermal growth factor receptor 2 was positively correlated with the expression of the vascular endothelial growth factor, further speculating that there may be a link between human epidermal growth factor receptor 2 and angiogenesis in metastatic colorectal cancer [21]. Simvastatin inhibits angiogenesis in human epidermal growth factor receptor 2+ colorectal cancer cells.

### 2.3. Simvastatin Can Enhance the Radiosensitivity of Colorectal Cancer Cells

Bass et al. (2015) used simvastatin, radiotherapy alone, and combined therapy on 3 patients with colorectal cancer, respectively, and then compared the curative effects of the 3 patients. The results found that simvastatin not only effectively reduced the vitality of colorectal cancer cells but also enhanced the sensitivity of cancer cells to radiation *in vitro* [22]. It is speculated that this may be related to the depletion of GGPP and the effected EGFR-RAS-ERK1/2 pathway, reducing the phosphorylation of extracellular signal-regulated kinases (ERK1/2) [23].

### 2.4. The Effect of Simvastatin on Cancer Stem Cells

Simvastatin can slow down the proliferation of cancer stem cells. Possibly, it is related to the fact that simvastatin inhibits the activity of DNMT, which in turn affects the two promitogenic signaling pathways PI3K/AKT and MEK/ERK in colorectal cancer [24]. However, some scholars believe that simvastatin, as an inhibitor of DNMT, can demethylate the promoter region of the bone morphogenetic protein (BMP), tissue inhibitor of metalloproteinase (TIMP3), and HIC-1 gene and can reactivate BMP to inhibit tumor stem cells and resensitize colorectal cancer cells to 5-Fu treatment [25].

### 2.5. Simvastatin-Induced Activation of Nrf2

Nuclear factor E2-related factor 2 (Nrf2) is a transcription factor that activates the intracellular antioxidant stress response. Simvastatin can affect the expression of Nrf2 through the ERK and PI3K/AKT pathways in HT-29 and HCT-116 colorectal cancer cells, thereby inducing the high expression of antioxidant enzymes, thereby inhibiting the proliferation of colorectal cancer cells.

RETRACTED

### 2.6. Simvastatin Upregulates GSK3*β* and Downregulates CDK4/Cyclin D1 and CDK2/Cyclin E1

The human cell cycle is regulated by the cyclic activation or inactivation of cyclin-dependent kinases (CDK) and their inhibitors, such as p21 and p27. Cyclins C1, D, and E bind to CDK4/6 and CDK2, respectively, and initiate the transition from the G1 phase to the S phase. Appropriate levels of cyclin D1 play a key role in the progression of the G1-S cell cycle transition. Glycogen synthase kinase 3*β* (GSK3*β*) is an important regulatory protein. Simvastatin upregulates GSK3*β* and inhibits CDK4/cyclin D1 and CDK2/cyclin E1, thereby blocking the cell cycle in the G1 phase in colorectal cancer.

### 2.7. Simvastatin Activates miR-192 to Inhibit Cancer Cell Proliferation

A novel tumor suppressor RNA miR-192 is an important endogenous biomolecule in the human body. Related studies have shown that miR-192 is overexpressed in colorectal cancer HCT-116 cells. Ras-associated protein Rab-2A (RAB2A) was bioinformatically identified as a downstream target of miR-192. Simvastatin, an activator of miR-192, upregulated its expression in colorectal cancer cells and acted on RAR2A to inhibit not only colon cancer cell proliferation but also to reduce *β*-catenin to inhibit epithelial-mesenchymal transition and thus cancer cell migration.

## 3. Exploration of Simvastatin in the Treatment of Colorectal Cancer

### 3.1. XELIRI/FOLFIRI Regimen Combined with Simvastatin

A total of 288 patients were recruited from 7 cancer hospitals in Japan, and a phase III clinical trial of XELIRI/FOLFIRI combined with simvastatin/placebo in colorectal cancer patients was carried out to explore whether this regimen provides a survival benefit in previously treated rectal cancer patients and to confirm progression-free survival [26]. Finally, the median progression-free survival in the study group and observation group was 6.1 months and 7.3 months, respectively, the median overall survival in the two groups was 15.7 months and 20.1 months, respectively, and there was an absence of statistical difference in the progression-free survival and overall survival in the two groups. Presumably, it is associated with the underdosing of the trial simvastatin. Simvastatin has a biphasic effect on angiogenesis. Simvastatin accelerates endothelial cell proliferation at low concentrations (0.005–0.01 *μ*mol/L); at high concentrations (0.05–1 *μ*mol/L), it inhibits endothelial cell proliferation, migration, and differentiation. Most preliminary clinical studies have used high doses of simvastatin that are not permitted for use in humans. Therefore, in this clinical trial, an accepted safe dose (40 mg/d) was used, but this dose may not be sufficient to inhibit tumour cell proliferation.

RETRACTED

### 3.2. CAPOX + Bevacizumab Regimen Combined with Simvastatin

Simvastatin is an antiangiogenic inhibitor that potentiates the effect of bevacizumab *in vitro* and *in vivo*. Previously, it is proved that simvastatin doses of 40 mg/d during chemotherapy may not have an anticancer effect. A phase III clinical trial was designed to evaluate the addition of simvastatin (80 mg/d) to CAPOX + bevacizumab regimen in the efficacy and safety of chemotherapy in patients with colorectal cancer. A total of 86 patients with colorectal cancer were recruited in this study, and all patients received standard CAPOX + bevacizumab chemotherapy and simvastatin (80 mg/d) was added during treatment. The results revealed that the median progression-free survival for all patients was 11.2 months, and the median overall survival was 18.7 months, and the disease control rate and overall response rate were 87.6% and 57.8%, respectively [27]. Progression-free survival results in this trial were more favourable compared to previous studies, with median overall survival results similar to those of CAPOX + bevacizumab alone. It was therefore concluded that the addition of simvastatin to CAPOX + bevacizumab chemotherapy prolonged progression-free survival in patients with colorectal cancer with no additional toxicity [28].

### 3.3. Trial of Simvastatin for an Adjuvant Therapy of Rectal Cancer

Radical resection of rectal cancer after adjuvant chemoradiotherapy is considered the standard treatment for locally advanced rectal cancer in the industry. Despite the ability to enhance the radiosensitivity of rectal cancer cells, a recent Chilean study found that the addition of simvastatin during adjuvant chemoradiotherapy failed to improve progression-free survival in patients with rectal cancer [29]. It is hypothesized that this is related to the inadequate daily dose of simvastatin, which affects long-term oncological outcomes [30]. More clinical trials are needed to verify whether simvastatin can be used in the adjuvant treatment of rectal cancer.

### 3.4. Analysis of Whether Simvastatin Can Reduce the Risk of Colorectal Cancer

Lee et al. (2015) found in an observational study that long-term (≥3 years) use of simvastatin is associated with a low risk of colorectal cancer [31]. A team at the University of Pennsylvania School of Medicine conducted a retrospective study and found that starting to administrate simvastatin at least 60 days before colonoscopy reduced the incidence of PC-CRC-3y by 31% [32]. However, critics have argued that most of these studies had less than 3 years of follow-up and that data on cancer incidence and mortality were also omitted from the randomized comparative trials of cardiovascular effects, inevitably leading to biased statistical results [33]. In view of this, the independent relationship between the risk of colorectal cancer, the use of simvastatin, and changes in serum cholesterol concentrations should be first clarified when analyzing whether simvastatin can reduce the risk of colorectal cancer. Zhang et al. (2009) conducted a subgroup analysis of the population who had previously received simvastatin and found that there was no significant difference in the risk of colorectal cancer among those who continued or stopped taking simvastatin, but the increase in serum cholesterol levels was independently associated with the risk reduction of colorectal cancer. We hypothesize that the idea that simvastatin reduces the risk of colorectal cancer in previous studies does not exclude the potential confounding effect of serum cholesterol prior to the use of simvastatin and that there may be concurrent use of simvastatin in people with a lower risk of cancer, which could lead to biased trial results and conclusions [34]. Clinical studies have confirmed that higher serum cholesterol levels can effectively reduce the risk of colorectal cancer. It raises a question for us that whether the recent unexplained drop in serum total cholesterol in the subject can indicate a risk of colorectal cancer [35]. To date, there are few studies on the relationship between cholesterol measurement time and colon cancer diagnosis, serum cholesterol changes, and colorectal cancer risk, and thus more clinical evidence is required to collaborate the hypothesis that simvastatin can reduce colorectal cancer risk.

RETRACTED

## 4. Conclusion

Colorectal cancer is a common malignant tumor of the digestive system and its incidence is second only to lung cancer in the global malignant tumor. Common clinical symptoms of colorectal cancer include blood in the stool, abdominal pain, weight loss, and intestinal obstruction [36]. The causes of colorectal cancer are generally considered to be the following: (1) the development of colorectal cancer is closely related to dietary factors, such as low-fibre diet, high-fat and high-protein diet, and lack of micronutrients and vitamins are all risk factors for colorectal cancer [37]; (2) genetic factors play an important role in the development of colorectal cancer. In addition, the risk of colorectal cancer is four times higher in people with a family history of colorectal cancer [38, 39]; and (3) nitrosamines and their compounds are the most important chemical carcinogens causing colorectal cancer, and methyl aromatic amines in fried and baked foods are also closely related to the development of colorectal cancer [40]. There are also parasites and lifestyle factors [41]. The mainstay for colorectal cancer includes surgery, drug therapy, and radiation therapy, of which surgical therapy is suitable for patients with carcinoma in situ and early-stage cancer. Regarding patients with advanced cancer, surgery remains less than satisfactory, and drugs and radiation are frequently combined [42]. Bevacizumab, cetuximab, and panitumumab are commonly used in chemoradiotherapy and drug therapy in clinical practice, and the rational therapy should be formulated, tailoring the specific conditions of patients [43].

Statins are a general term for a class of lipid-lowering drugs that have been used in many other diseases in addition to their promising use in colorectal cancer. Lovastatin has the effect of lowering total cholesterol and LDL cholesterol and can be used to modulate lipids in the treatment of patients with primary hypercholesterolaemia [44]; fluvastatin is often used in the treatment of patients with primary hypercholesterolaemia for lipid modulation, which helps to reduce lipid levels and in patients with mixed dyslipidaemia [45]; atorvastatin is used as a lipid-modifying drug, which can be applied in the treatment of hypercholesterolaemia when nonpharmaceuticals are not effective, and also in the treatment of coronary artery diseases [46]. In recent years, numerous scholars believe that simvastatin has the potential to treat colorectal cancer, and many clinical studies have confirmed that simvastatin realizes clinical anticancer effects by inhibiting the proliferation and migration of endothelial cells and inducing apoptosis [47]. In the dimension of drug reuse, simvastatin exhibits a good anticancer potential. Its anticancer effect in preclinical research has prompted scholars to explore its use as a cancer treatment drug; also, many related studies have confirmed the feasibility of the drug, yet further clinical studies are still needed to confirm its outcome [48]. Notably, the adverse effects of simvastatin are of concern as long-term administration of simvastatin may cause symptoms such as rhabdomyolysis and hepatotoxicity [49]. In view of this, the optimal clinical dose and duration of use needs to be determined to ensure patient safety [31, 50, 51].

RETRACTED

There are few clinical studies on the treatment of colorectal cancer patients with simvastatin, and the specific mechanism of action of simvastatin in the treatment of colorectal cancer has not been studied in depth at multiple levels. Obviously, the most important work at present is to identify the molecular mechanism of the antitumor effect of simvastatin, which includes the specific effects, pathways and targets of each mechanism, such as the mechanism of inhibiting tumor angiogenesis. This rules out controversy about the antitumour effects of simvastatin analogues and proves them at the protein and genetic level. A full understanding of the sensitivity of simvastatin to tumour cells and the specific pathways of action of simvastatin cytotoxicity will help to reveal new molecular targets for simvastatin in the treatment of colorectal cancer and help to explore the maximisation of its efficacy, maximum tolerated dose, and toxicity. Clinical applications [52]. We look forward to more reports on the application of simvastatin in the treatment of colorectal cancer in the future.

## Data Availability

The datasets used and analysed during the current study are available from the corresponding author on reasonable request.
